# Machine Learning for Diagnosis of Systemic Lupus Erythematosus: A Systematic Review and Meta-Analysis

This article has been retracted.

**DOI:** 10.1155/2022/7167066

**Published:** 2022-11-22

**Authors:** Yuan Zhou, Meng Wang, Shasha Zhao, Yan Yan

**Affiliations:** Department of Dermatology, Plastic Surgery Hospital, Chinese Academy of Medical Sciences and Peking Union Medical College, Beijing, China

## Abstract

**Background:**

Application of machine learning (ML) for identification of systemic lupus erythematosus (SLE) has been recently drawing increasing attention, while there is still lack of evidence-based support.

**Methods:**

Systematic review and meta-analysis are conducted to evaluate its diagnostic accuracy and application prospect. PubMed, Embase, Cochrane Library, and Web of Science libraries are searched, in combination with manual searching and literature retrospection, for studies regarding machine learning for identifying SLE and neuropsychiatric systemic lupus erythematosus (NPSLE). Quality Assessment of Diagnostic Accuracy Studies (QUADA-2) is applied to assess the quality of included studies. Diagnostic accuracy of the SLE model and NPSLE model is assessed using the bivariate fixed-effect model, and the data are pooled. Summary receiver operator characteristic curve (SROC) is plotted, and area under the curve (AUC) is calculated.

**Results:**

Eighteen (18) studies are included, in which ten (10) focused on SLE and eight (8) on NPSLE. The AUC of SLE identification is 0.95, the sensitivity is 0.90, the specificity is 0.89, the PLR is 8.4, the NLR is 0.12, and the DOR is 73. AUC of NPSLE identification is 0.89, the sensitivity is 0.83, the specificity is 0.83, the PLR is 5.0, the NLR is 0.20, and the DOR is 25.

**Conclusion:**

Machine learning presented remarkable performance in identification of SLE and NPSLE. Based on the convenience for inclusion factor collection and non-invasiveness of detection, machine learning is expected to be widely applied in clinical practice to assist medical decision making.

## 1. Introduction

Systemic lupus erythematosus (SLE) is an autoimmunity-mediated, chronic, and refractory connective tissue disease (CTD) with multiple systems involved. It usually occurs in women aged 20 to 40 years old, and the ratio of incidence between male and female is 1 : 9. The prevalence of PLE varies from 1 to 10 per 100000 people in different countries and regions, and the incidence in coloured people is higher than that in white people [1–3].

Commonly used clinical diagnostic criteria included American College of Rheumatology (ACR) criteria [4], Systemic Lupus International Collaborating Clinics (SLICC) criteria [5], and European League Against Rheumatism/American College of Rheumatology Classification (EULAR/ACR) Criteria [6] for Systemic Lupus Erythematosus. Sensitivity and specificity reported in different cohorts range from 0.84 to 0.95 [7]. However, early identification and diagnosis for SLE are still difficult due to the heterogeneity of its clinical and laboratorial indicators. The multiple organ damage would aggravate over time, making early recognition and diagnosis of SLE important [8]. Diagnosis of neuropsychiatric systemic lupus erythematosus (NPSLE) currently follows the ACR criteria [9], which is mainly based on clinical symptoms that have already occurred, and occurrence of those symptoms typically indicates highly active NPSLE with high mortality, presenting a challenge to the early identification for NPSLE. Machine learning (ML) refers to a technology to make computer simulate or implement human learning activities, which can make full use of information via algorithms to obtain hidden, effective, and understandable knowledge from massive data, so as to build predictive models [10]. Recently, ML has shown excellent pattern-recognizing capability and has gradually affected clinical decision making in multiple fields, including rheumatic immunology [11, 12].

Its value for SLE and NPSLE identification and diagnosis is particularly brought into focus. However, the diagnostic accuracy varies in different models, and there is also lack of evidence-based support. We conducted this meta-analysis to identify the value of machine learning in the recognition of SLE and NPSLE and to explore which predictors are more clinically significant, so as to provide reference for future development of diagnostic systems and models.

## 2. Methods

The systematic review and meta-analysis were conducted in strict accordance with the Preferred Reporting Items for Systematic Reviews and Meta-Analyses (PRISMA) [13] statement and had been registered on PROSPERO (registration no. CRD42022329180).

### 2.1. Definition

In this study, SLE is defined as patients meeting the ACR [4] or SLICC [5] criteria, and NPSLE is defined as patients meeting the NPSLE ACR [9] criteria.

### 2.2. Hypothesis

Can machine learning applications play a significant role in the identification of systemic lupus erythematosus (SLE) and neuropsychiatric systemic lupus erythematosus (NPSLE)?

### 2.3. Literature Search and Study Selection

PubMed, Embase, Cochrane Library, and Web of Science were searched from inception to March 2022, via combination of medical subject headings and free words, for studies that applied ML for identification of SLE and NPSLE. Manual searching and literature retrospection were also conducted. Search items in PubMed included “Lupus Erythematosus, Systemic,” “Systemic Lupus Erythematosus,” “Lupus Erythematosus Disseminatus,” “Libman-Sacks Disease,” “machine learning,” “Deep learning,” “Transfer Learning,” “Ensemble Learning,” “artificial intelligence,” and “Prediction model,” with the language restricted to English.

Patients who have symptoms of SLE or NPSLE were included. Exclusion criteria were as follows:

1. Patients who had history of other cerebral diseases.
2. Unable to participate in relevant clinical and laboratory tests.
3. Concomitant with other CTDs. Eligible randomized controlled trails (RCTs), case-control studies, cross-sectional studies, nested case-control studies, and cohort studies were all included.
4. Studies with the participants less than 30 in training set of the model or without modeling were excluded.

### 2.4. Literature Screening and Data Extraction

All identified articles were imported to Endnote. The titles and abstracts were browsed following duplicate removal to exclude irrelevant studies. Full texts of the remaining articles were read, according to the inclusion and exclusion criteria, to screen out eligible studies. Extracted data included name of first author, publication date, sample size, types of models, indices of modeling, and outcome measures. Outcome measures included sensitivity (SEN), specificity (SPE), positive likelihood ratio (PLR), negative likelihood ratio (NLR), diagnostic odds ratio (DOR), summary receiver operator characteristic curve (SROC), area under the curve (AUC), and clinical application value. Literature screening and data extraction were conducted by two reviewers (Yuan Zhou and Meng Wang) independently, and any disagreements were settled via discussion with a third reviewer (Shasha Zhao).

### 2.5. Quality Assessment

Quality assessment of included studies was performed by two reviewers using Quality Assessment of Diagnostic Accuracy Studies (QUADAS-2) criteria [14], which contain four (4) domains in terms of risk of bias: patient selection, index test, reference standard, and flow and timing. Each domain was assessed, and the results were pooled to grade an included study as “low risk,” “high risk,” or “unclear risk.” Disagreements were resolved by a third reviewer to reach a consensus.

### 2.6. Statistical Analysis

Statistical analysis was performed using STATA 15.0. A grouping analysis was processed based on different types of machine learning algorithms. C-indices with 95% confidence intervals (95% Cis) of the prediction models were pooled. Then, the diagnostic accuracy of ML for SLE and NPSLE was evaluated using the bivariate fixed-effect model. Outcomes that were included in the model contained point-estimated values of SEN, SPE, PLR, NLR, and DOR, with their 95% CIs provided. The SROC was plotted, and AUC with its 95% CI was calculated. Deek's funnel plot was applied to assess the publication bias, and *Q* and *I*^2^ statistics were used for heterogeneity test. *I*^2^ greater than 50% indicated significant heterogeneity. *p* value less than 0.05 indicated statistical significance.

## 3. Results

### 3.1. Study Selection and Risk of Bias Assessment

Sixteen hundred and eighty-one (1681) articles were identified through initial search, and 1226 remained after removing duplicates. Eleven hundred and sixty-six (1166) ineligible articles were excluded after browsing the abstracts and titles, and full texts of the remaining sixty (60) articles were read. Finally, a total of eighteen (18) studies were included, in which ten (10) [15–24] focused on SLE and the remaining eight (8) [25–32] on NPSLE. The study selection process is shown in Figure 1, and the characteristics of included studies are shown in Tables 1 (for SLE) and 2 (for NPSLE). Among the eighteen (18) studies, fifteen (15) were published in recent five (5) years, and thirteen (13) were published in recent three (3) years, which revealed that this field might be an emerging hotspot and innovative.

Risk of bias assessment for included studies was conducted according to QUADAS-2 criteria, via RevMan 5.3 software. The results are shown in Figure 2.

High risk of bias might be inevitable because most of the included studies (*n* = 13) were retrospective case-control design studies, and studies on NPSLE had limited sample size. Clinical practicability of included studies was graded as low risk, suggesting considerable clinical value of our study. We divided the included studies into a SLE subgroup and NPSLE subgroup for heterogeneity test and publication bias assessment, as shown in Figures 3 and 4, respectively.

### 3.2. Diagnostic Performance of ML for SLE

There are 10 studies included in meta-analysis for ML in SLE identification, with 15 different models and 19631 participants. Among the studies, 5 are from registration databases and 5 from retrospective case-control studies, with sufficient sample size. The results of analysis are presented in Figures 5(a), 6(a), 7(a), and 8(a). The AUC is 0.95 [95% CI (0.93, 0.93)], the sensitivity is 0.90 [95% CI (0.85, 0.93)], the specificity is 0.89 [95% CI (0.86, 0.92)], the PLR is 8.4 [95% CI (6.2, 11.4)], the NLR is 0.12 [95% CI (0.08, 0.17)], and the DOR is 73 [95% CI (40–134)]. According to Figure 7(a), based on a hypothesis of PLR = 10 and NLR = 0.1, there are still 8 algorithms that could competently distinguish SLE patients and non-SLE patients, in which 3 algorithms are in critical state.  Figure 8 reveals the post-test probability of ML for SLE diagnosis, which indicated that assuming that the pre-test probability is 50%, the post-test probability of ML for SLE diagnosis is 0.89, and the probability of being diagnosed as non-SLE is 0.1.

### 3.3. Diagnostic Performance of ML for NPSLE

There are 8 studies included in meta-analysis for ML in NPSLE identification, with 18 different models and 569 participants. All the studies are from retrospective case-control studies, with limited sample size. The results of analysis are presented in Figures 5(b), 6(b), 7(b), and 8(b). The AUC of NPSLE identification is 0.89 [95% CI (0.86, 0.92)], the sensitivity is 0.83 [95% CI (0.79, 0.87)], the specificity is 0.83 [95% CI (0.76, 0.88)], the PLR is 5.0 [95% CI (3.4, 7.3)], the NLR is 0.20 [95% CI (0.15, 0.27)], and the DOR is 25 [95% CI (13–47)]. Based on a hypothesis that PLR = 10 and NLR = 0.1, there are 3 ML models that could competently distinguish NPSLE patients and non-NPSLE patients. ML also presented excellent diagnostic performance for NPSLE.

## 4. Discussion

In this study, we reviewed studies that applied ML to diagnose SLE and NPSLE and conducted a meta-analysis. This is the first meta-analysis performed to evaluate the performance of ML for SLE identification, with high clinical significance. ML is the combination of statistics and computer science, which can make full use of information and obtain veiled, effective, and understandable knowledge from massive data to reveal connections between the data so as to build prediction models. ML typically falls into two categories: supervised learning and unsupervised learning [33–35]. It can assist clinicians in decision making via its remarkable pattern-recognizing capability and has shown excellent performance in identification for inflammatory diseases, cardiovascular diseases, and brain diseases [36, 37].

There are various ML models designed for SLE, with sufficient participants. Types of the models did not affect the diagnostic accuracy. Commonly applied methods such as random forest (RF) and logistic regression (LR) are used because most of the models included more than 10 variables. RF could produce highly accurate classifiers for various types of data and could evaluate the importance of variables when determining categories, so that it could produce unbiased estimates for generalized errors [38, 39]. This could relatively ensure the accuracy of multivariate modeling. LR is a machine learning method designed to solve classification problems. It is a predictive analysis based on probability distribution [40]. LR is less likely to overfit, although that might occur in high-dimensional datasets. The training time of LR is shorter than that of most complex algorithms (such as artificial neural network) due to the simplicity of probability interpretation; therefore, it has relatively practical diagnostic performance [41, 42]. The rest of the models, such as SVM, DT, and ANN, are also applied, with comparatively remarkable diagnostic performance. Among the 10 studies, 8 used K-fold cross validation and 8 used external validation. Accuracy of the models is reliable. Most of the models included clinical and laboratorial data as variables and added extra variables on the basis of ACR, EULAR, and SLICC criteria. The risk factors are ordered based on the model itself, which provided more directions and basis for us to improve the SLE classification criteria. On the other hand, there are 3 studies [20, 22, 23] that performed analyses for blood polypeptides and lipids, and 1 study [21] distinguished SLE patients from normal people through skin imaging examination. All of these studies yielded decent results and provided more directions for early identification of SLE in clinical practice.

There are limited number of studies that focused on ML for NPSLE, and MRI results are applied in these studies for learning and modeling so that most of the studies applied support vector machine (SVM) [43, 44]. ML has been widely applied in imaging diagnosis for many diseases such as brain metastases, retinopathy, and so on and has been statistically validated by meta-analysis [45, 46]. The optimization of SVM takes into account the minimization of empirical risk and structural risk so that it is stable. From a geometric point of view, the stability of SVM is reflected in that it requires the largest margin when constructing a hyperplane decision boundary; therefore, there is plenty of space between the boundaries to contain test samples, which is more suitable for solving image problems [47]. There are 5 studies that applied K-fold cross validation and 4 studies that applied external validation to improve accuracy of the models, and SVM tended to overfit when the sample size was too small. Xiao et al. compared the results of ML with those of two senior radiologists and found the former to be more competent, which further improved the efficacy of ML. However, in the model training process, hundreds of different brain functional areas need to be identified and analyzed one by one, and then are sorted by the degree of influence, and the parts with greater influence are selected for modeling, which often requires long time of training. With the wide and deep application of ML in imaging, it is necessary to improve the algorithm, increase the training efficiency, and reduce the time of training.

It is worth mentioning that in the process of searching the literature, we found that there are a large number of studies based on molecular and genetic levels, using machine learning methods to identify SLE risk genes or SLE-related antibodies. [48–55]. Several studies applied ML to evaluate the activity and prognosis of SLE [56–61] and to assist in classification of lupus nephritis [62, 63]. All these studies yielded satisfying results. Apart from all these, systematic literature reviews have been applied in different fields, such as rough set exploration system [64], machine learning methods for cyber security [65], and meta-learning for algorithm selection [66]. To sum up, ML is expected to play a variety of roles in clinical practice, and more relevant studies are needed.

### 4.1. Limitations

Though a comprehensive search was conducted in PubMed, Embase, Cochrane, and Web of Science, the number of included studies is small. Secondly, there is significant heterogeneity among the studies in terms of variable selection. We look forward to including more clinically significant, noninvasive, and easily collectible variables to further refine the model. At the same time, studies that focused on ML for NPSLE had limited sample size. It is difficult to recruit patients in countries with small populations so that most of the studies are from China, leading to lack of multiracial comparison. However, as NPSLE clinically represents the high activity and lethality of SLE, it is useful and necessary to conduct relevant meta-analysis. More ML models are needed to identify NPSLE in different races. Lastly, due to the clinical practice and the nature of the diagnostic experiment itself, the literatures included in this study inevitably lack prospective studies.

## 5. Conclusion

Machine learning (ML) is expected to be widely applied in clinical practice to assist in medical decision making. ML techniques can be used for the identification of systemic lupus erythematosus (SLE) and neuropsychiatric systemic lupus erythematosus (NPSLE). These techniques are considered an effective auxiliary method for the diagnosis of these diseases. These techniques gained great attention of the researchers, but there is still lack of evidence-based support. Systematic review and meta-analysis were conducted to evaluate the diagnostic accuracy and application prospect of ML techniques. Four libraries (PubMed, Embase, Cochrane Library, and Web of Science) were searched for the collection of relevant articles regarding machine learning for identification or diagnosis of SLE and NPSLE. Diagnostic accuracy of the SLE and NPSLE models was assessed using the bivariate fixed-effect model. Out of eighteen (18) studies, ten (10) were related to SLE and eight (8) to NPSLE. The AUC of SLE identification is 0.95, the sensitivity is 0.90, and the specificity is 0.89. AUC of NPSLE identification is 0.89, the sensitivity is 0.83, and the specificity is 0.83. It is concluded that ML played a significant role in identification of SLE and NPSLE.

## Figures and Tables

**Figure 1:** Flowchart of the identification, inclusion, and exclusion of studies.

**Figure 2:** Quality evaluation of the included literature.

**Figure 3:** Heterogeneity analysis: (a) for SLE; (b) for NPSLE.

**Figure 4:** Publication bias: (a) for SLE; (b) for NPSLE.

**Figure 5:** Diagnostic performance of machine learning: (a) for SLE; (b) for NPSLE.

**Figure 6:** The summary receiver operating characteristic (SROC) curve for the diagnostic performance of machine learning: (a) for SLE; (b) for NPSLE.

**Figure 7:** Likelihood matrix diagram of clinical application of machine learning: (a) for SLE; (b) for NPSLE.

**Figure 8:** Fagan's diagram of the clinical application of machine learning: (a) for SLE; (b) for NPSLE.

**Table 1:** Characteristics of the included studies for SLE.

Author	Year	Country	Sample	Prediction	Definition	Sample number of training set (event/all)	K-fold cross validation	External validation	Model
Murray et al.	2019	USA	Registration data	Diagnosis	ACR	583/16767	10	Yes	LR
Ceccarelli et al.	2021	Italy	Case-control	Diagnosis	EULAR/ACR	173/306	No	NA	LR, SVM, DT
Barnado et al.	2022	USA	Registration data	Diagnosis	NA	121/249	5	Yes	RF, XGB
Jorge et al.	2019	USA	Registration data	Diagnosis	ACR/SLICC	66/200	No	Yes	LR
Adamichou et al.	2020	Greece	Registration data	Diagnosis	NA	401/802	10	Yes	LR
Huang et al.	2009	China	Case-control	Diagnosis	ACR	32/118	No	Yes	DT
Samundeswari et al.	2018	India	Case-control	Diagnosis	ACR	200/400	10	NA	ANN, SVM
Dai et al.	2010	China	Case-control	Diagnosis	ACR	50/99	10	Yes	KNN
Matthiesen et al.	2021	Portugal	Case-control	Diagnosis	NA	64/128	10	Yes	PLS
Turner et al.	2017	USA	Registration data	Diagnosis	ACR	272/562	5	Yes	ANN, RF, NB, SVM, Word2Vec

**Table 2:** Characteristics of the included studies for NPSLE.

Author	Year	Country	Sample	Prediction	Definition	Sample number of training set (event/all)	K-fold cross validation	External validation	Model	MRI machine	Tesla	Slice thickness (mm)
Tan et al.	2021	China	Case-control	Diagnosis	ACR	23/39	10	NA	Bagging, DT, SVM, AdaBoost, PCA + AdaBoost, VAE + SVM, PCA + DT, PCA + bagging, PCA + SVM, GA + SVM, MARL + GA + SVM	NA	3	NA
Li et al.	2020	China	Case-control	Diagnosis	ACR	23/39	3	NA	BL-SVM	SIGNA, General Electric Medical Systems	3	5
Zhuo et al.	2019	China	Case-control	Diagnosis	ACR	31/63	Leave-one-out CV	NA	SVM	Non-invasive 3D ASL-MRI; GE MR750, GE Healthcare	3	NA
Sun et al.	2010	China	Case-control	Diagnosis	ACR	27/54	NA	Yes	Decision tree	NA	NA	NA
Simos et al.	2019	Greece	Case-control	Diagnosis	EULAR	41/72	5	NA	SVM	Resting-state fMRI, Siemens Vision/Sonata scanner (Erlangen, Germany)	1.5	3
Inglese et al.	2022	Netherlands	Case-control	Diagnosis	ACR	68/136	NA	Yes	SVM	Philips Healthcare, Best, Netherlands	3	NA
Luo et al.	2022	China	Case-control	Diagnosis	ACR	36/83	NA	Yes	SVM	MAGNETOM Verio scanner (Siemens Healthcare)	3	6
Simos et al.	2020	Greece	Case-control	Diagnosis	EULAR	44/83	5	Yes	Random forest	Resting-state functional MRI, (Vision/Sonata, Siemens/Erlangen)	1.5	3

## Data Availability

The datasets used during the current study are available from the corresponding author on reasonable request.
